This article has been retracted.

# Proteomics Approaches for Identification of Tumor Relevant Protein Targets in Pulmonary Squamous Cell Carcinoma by 2D-DIGE-MS

**DOI:** 10.1371/journal.pone.0095121

**Published:** 2014-04-16

**Authors:** Hao Lihong, Gong Linlin, Guo Yiping, Song Yang, Qi Xiaoyu, Guan Zhuzhu, Yang Xiaohan, Zhou Xin, Xue Liyan, Shao Shujuan

**Affiliations:** 1 Key Laboratory of Proteomics, Dalian Medical University, Dalian, Liaoning Province, P.R. China; 2 Department of Pathology, Cancer Institute and Hospital, Chinese Academy of Medical Sciences (CAMS) and Peking Union Medical College (PUMC), Beijing, P.R. China; Vanderbilt University Medical Center, United States of America

## Abstract

Potential markers for progression of pulmonary squamous cell carcinoma (SCC) were identified by examining samples of lung SCC and adjacent normal tissues using a combination of fluorescence two-dimensional difference gel electrophoresis (2D-DIGE), matrix-assisted laser desorption/ionization time of flight mass spectrometry (MALDI-TOF-MS), and electrospray ionization quadrupole-time of flight mass spectrometry (ESI-Q-TOF). The PANTHER System was used for gel image based quantification and statistical analysis. An analysis of proteomic data revealed that 323 protein spots showed significantly different levels of expression (P≤0.05) in lung SCC tissue compared to expression in normal lung tissue. A further analysis of these protein spots by MALDI-TOF-MS identified 81 different proteins. A systems biology approach was used to map these proteins to major pathways involved in numerous cellular processes, including localization, transport, cellular component organization, apoptosis, and reproduction. Additionally, the expression of several proteins in lung SCC and normal tissues was examined using immunohistochemistry and western blot. The functions of individual proteins are being further investigated and validated, and the results might provide new insights into the mechanism of lung SCC progression, potentially leading to the design of novel diagnostic and therapeutic strategies.

## Introduction

Lung cancer is the leading cancer-related cause of death worldwide in both men and women. In China, the mortality rate for lung cancer has increased by 465% during the last 30 years, making it the most deadly of all malignant tumors. Despite advances in treatments such as surgery, chemotherapy and radiotherapy, the clinical prognosis for patients with lung cancer remains poor, and the overall 5-year survival rate is only 10-15% [1]. This is because at the time of diagnosis, most lung cancer patients present with an advanced stage of disease. Therefore, there is an urgent need to identify biomarkers that are useful for detection of early-stage lung cancer, and developing a prognosis for long-term survival of patients. Recently, novel technology linked to development of the human genome database, e.g. proteomics, has been utilized to identify protein biomarkers associated with tumor development and progression. Two-dimensional differential in-gel electrophoresis [2]–[5] (2D-DIGE), is an advanced quantitative proteomics technology which offers higher sensitivity, accuracy, and resolution compared with traditional two-dimensional polyacrylamide gel electrophoresis (2-DE). This method is used to pre-label different protein samples with fluorescent cyanine dyes (Cy2, Cy3, and Cy5) prior to separation by 2-DE. Therefore, different samples can be labeled with different dyes and separated in the same 2D gel; also, the same internal standard can be used in every gel so as to avoid intergel variation. Thus, 2D-DIGE can be used to obtain an accurate and reproducible quantitation of differences between samples [4].

In the present study, we investigated the proteome of pulmonary squamous cell carcinoma, and compared its profile to that of adjacent histologically normal tissue by using a 2-D differential in-gel electrophoresis (2D-DIGE) system for protein 2-D electrophoresis [5], matrix-assisted laser desorption/ionization time of flight mass spectrometry (MALDI-TOF-MS), and electrospray ionization quadrupole-time of flight mass spectrometry (ESI-Q-TOF) for protein identification. The differentially expressed proteins were analyzed using bioinformatic approaches, and further validated by western blot and immunohistochemical (IHC) assays. The goal of our study was to identify differentially expressed proteins that could serve as novel biomarkers for lung cancer. Although the proteomics profile of non-small cell lung cancer (NSCLC) tissue has been previously reported [6]–[9], due it's the variability and low reproducibility of the findings, no final conclusions had yet been reached until now. In this study, we used samples of human clinical cancer tissue to investigate the protein profile of SCC tumors. Our results identified 81 differentially expressed proteins, 19 of which are been linked to lung cancer for the first time by our research group, and 9 novel proteins which had not been previously reported. Our results provide important supplemental data in the area of cancer proteomics.

## Material and Methods

### Clinical Samples

The protocol for this study was approved by the Medical Ethical Committee of Dalian Medical University, China, and all tissue samples and patient data were obtained after receiving written informed consent. Whole tissue samples used for analysis of protein expression were collected during surgeries performed on patients (6 males and 1 female) aged 36 to 67 years in the Department of Thoracic Surgery at the First Affiliated Hospital of Dalian Medical University from 2004 to 2006. The patients had not received preoperative therapy for their disease. Lung SCC samples and paired samples of adjacent normal bronchial epithelial tissue were removed, immediately placed in liquid nitrogen, and stored at −80°C.Tissue samples used for tumor classification were fixed in formalin and embedded in paraffin. Then, 5 µm frozen sections prepared from tissue blocks were briefly placed in ethanol, stained with hematoxylin and eosin, and subsequently histologically analyzed by a pathologist. Pathological staging was determined according to the latest TNM-classification system [10], and tumor grading was done according to Fuhrman [11]. Additionally, 20 pairs of SCC and adjacent normal tissue samples were subjected to western blot, and 104 samples of lung cancer tissue and 25 samples of normal tissue were subjected to IHC analysis. These samples were obtained from 44 female and 60 male volunteers (age range: 28–84 years, mean: 61 years) with different stages (20 with stage I, 34 with stage II, 50 with stage III) and grades (14 with G III, 47 with G II, and 43 with G I) of disease.

Serum samples for ELISA analysis were obtained from the Department of Thoracic Surgery at the First Affiliated Hospital of Dalian Medical University in 2013. These samples were obtained from a total of 150 lung cancer cases, which included 35 squamous cell carcinoma patients, 110 adenocarcinoma patients, 4 small cell carcinoma patients, and 1 polymorphic cell carcinoma patient, as well as 150 healthy donors. None of these patients had received preoperative therapy.

### Protein isolation

Proteins were isolated as described by Yu, LR [12]. Frozen tissue samples (50 g) were ground into fine powder on ice and homogenized in 300 µL of lysis buffer (Tris 30 mM, thiourea 2 M, urea 7 M, CHAPS 4% w/v, proteinase inhibitors 20 µL). The ground tissues samples were then solubilized by sonication (GE Healthcare Life Sciences, USA) on ice for 1 min and centrifuged at 12,000 rpm for 10 min at 4°C. Foreign substances were removed from the protein containing supernatant fractions (100 µL) according to a protocol included with a Clean-up kit. Total protein concentrations were determined using a quantitative 2D-Quant kit (GE Healthcare Life Sciences), and supernatant fractions were stored at −80°C.

### Cy-dye labeling

The pH value of each supernatant sample was adjusted to 8.5 by addition of 50 mmol/L NaOH. Then, 50 µg samples of lung SCC and paired normal sample lysates were labeled with Cy3 (500 pmol) and Cy5 (500 pmol), respectively. A mixture containing equal amounts of each protein sample was labeled with Cy2, and served as an internal standard to reduce intergel variation. Samples were reverse-labeled to eliminate both sample-dependent and dye-dependent bias. The labeling process was carried out in the dark and on ice for 30 min, and terminated by addition and reaction with 10 nmol lysine for 10 min under the same conditions.

### 2D-DIGE

Aliquots containing 150 µg of unlabelled protein pooled from equal amounts of samples were mixed with the Cy-dye labeled proteins described above. The mixtures were filled to a final volume of 450 µL by addition of a 2-fold volume of same buffer (2% carrier ampholyte 3–10, 2% DTT, 8 mol/L urea, 4% CHAPS, 2% IPG buffer) and IPG rehydration buffer (20 mmol/L DTT, 8 mol/L urea, 2% CHAPS, 1% IP buffer). After rehydration overnight, isoelectric focusing was carried out for a total of 74.5 kVhr. Subsequently, the IPG strips were soaked in 20 mL of solution A (6 mol/L urea, 50 mmol/L Tris-HCI, 30% glycerol, 2% SDS, 0.5% DTT, pH = 8.0) for 10 min for the first step of equilibration, and then soaked in 20 mL of solution B (0.5% DTT in solution A was replaced by 4.5% IAM (iodoacetamide)) for 10 min for the second step of equilibration, with both steps being protected from light. The strips were then placed on vertical SDS-PAGE gels and fixed with 12.5% agarose. SDS-PAGE was carried out using the Ettan DALT Six Electrophoresis System (GE Healthcare, Life Sciences, USA).

### Scanning and image analysis

The DIGE gels were scanned using a Typhoon TRIO laser scanner (GE Health Care Life Sciences). The excitation and emission wavelengths for Cy2, Cy3 and Cy5 were 488 nm and 520 nm, 532 nm and 580 nm, and 633 nm and 670 nm, respectively. The images of protein spots in each gel were detected, quantified, and normalized for intensity by analysis using DeCyder Differential Analysis software 5.0 (GE Healthcare Life Sciences). A differential in-gel analysis (DIA) module was used to detect the merged images of Cy2, Cy3, and Cy5 on each gel, while a biological variation analysis (BVA) module was used to automatically match all protein-spot maps. The student's t-test was used to assess the statistical significance of differences between differentially expressed proteins. Based on an average spot volume ratio, spots whose relative expression was changed ≥1.5-fold (increase or decrease) at the 95% confidence level (t-test; P<0.05) by representing a protein associated with a state of non-malignancy or malignancy were considered to be significant. The coordinates of significant spots were transferred to Deep Purple stained preparative gels for selection of spots for analysis by mass spectrometry.

### Mass spectrometry

Protein spots were cut from a preparative gel, in-gel digested with trypsin, and extracted as previously described [13]. C_18_-ZipTips (Millipore Billerica MA, USA) were used for MALDI target preparation according to the manufacturer's instructions. The concentrated and desalted peptides were eluted onto the MALDI target with CHCA matrix solution. Samples were analyzed to obtain their peptide mass fingerprint (PMF). The PMF spectra were processed using the DataExPlore software provided with the equipment, and the generated data were subsequently analyzed using the Mascot database (http://prospector.ucsf) and Profound database (http://129.85.19.192/profoundbin/WebProFound.exe). The following database search parameters were selected: the spectra were recorded in a mass range of 800 to 4000 Da; the error range of the apparent isoelectric point was ±0.5 pH; the error range of the apparent molecular weight was ±20%; fixed cysteine modification with carbamidomethyl; samples were derived from human beings; allowed non-restriction sites was 1; minimum matching peptide fragments was 5; trypsin fragments were run with a mass tolerance of 200 ppm; mass values were MH+. The proteins were determined based on the search results and the Ip and MW values in the gel.

### Bioinformatics analysis of proteomic data

For protein identification, peak lists were correlated with the PANTHER database [14] (http://www.pantherdb.org/) using the MF pie chart, CC pie chart, PC pie chart, and Pathway pie chart for analysis.

### Western blot

Samples of lung SCC tissue (50 mg) and paired normal tissue were lysed in 300 µL protein lysis buffer containing PMSF (100∶1) on ice, and then centrifuged at 12,000 rpm for 20 min at 4°C. Supernatant samples containing 50 µg of protein were separated by 12% SDS-PAGE gels and then transferred onto a nitrocellulose membrane. The membranes were blocked with 5% defatted milk for 1 h at room temperature, and then incubated with primary antibody rabbit anti-human SAP polyclonal antibody 1∶1000 (Abcam Cambridge MA, USA), mouse anti-human apoA1 polyclonal antibody 1∶500, and mouse anti-human actin monoclonal antibody 1∶3000 (Proteintech Group Inc. Chicago IL, USA) overnight at 4°C. Excess antibodies were removed by washing with TBST. Incubation with secondary antibodies (anti-mouse 1∶2000, anti-rabbit 1∶2000) was performed for 1 h at 37°C. The signals were detected using the electrogenerated chemiluminescence (ECL) visualization method, and the emitted light was captured by a Labwork gel imaging system (Bio-Rad Hercules CA, USA).

### Immunohistochemistry

Paraffin embedded tissue sections were dried overnight at 60°C, deparaffinized in xylene, and rehydrated through graded alcohols into water. Endogenous peroxidase activity was blocked by incubation with 3% hydrogen peroxide for 10 min. Microwave antigen retrieval was performed using EDTA for 20 min at temperatures of 65∼98°C in a microwave oven. Goat serum was used as the blocking reagent for 10 min at room temperature. The sections were incubated with primary antibody (rabbit anti-human SAP polyclonal antibody 1∶1000 (Abcam), rabbit anti-human apoA1 polyclonal antibody 1∶1000 (Proteintech Group, Inc.)) overnight at 4°C. Biotinylated secondary antibody and horseradish peroxidase-conjugated antibody were added for 20 min at room temperature and stained by DAB (ZSGB-BIO; Beijing, China) reagent for 5 min. Tissues used as negative controls were subjected to distilled water washing, hematoxylin counterstaining, dehydration, mounting, and PBS exposure instead of staining with a primary antibody.

### Enzyme-linked immunosorbent assay (ELISA)

Limosis blood was collected from a peripheral vein of each subject and centrifuged at 1500 rpm and 4°C for 10 min within 1 hour of collection; the obtained serum samples were stored at −80°C. Serum levels of apoA1 and SAP were measured by ELISA using a commercially available kit (Wuhan Huamei Biological Engineering Company Limited, China). Serum sample OD values were measured at 450 nm using a microplate reader (Thermo, USA) within 15 min to calculate the concentrations of apoA1 and SAP.

### Statistical Analysis

Differences between groups were evaluated using SPSS software. All comparisons were two-tailed, and P-values <0.05 were considered statistically significant.

## Results

### 2D-DIGE proteome map

The proteomes of pulmonary SCCs obtained from 7 cancer patients and paired normal tissues were analyzed by 2D-DIGE in a nonlinear pI range of 3.0–10.0 and a molecular weight range of 10 to 120 kDa. To systematically compare the performance of different staining methods used in differential protein profiling, a DIGE gel was run with an independently prepared proteome from a paired normal tissue stained with Cy3 (green), from SCC tissue stained with Cy5 (red), and from a mixture of all protein samples as the internal standard stained with Cy2 (blue). The black-and-white scanning images of each stained gel were showed at right (Figure 1). The digital images were analyzed using DeCyder software. A total of 323 spots were significantly altered in their abundance (P≤0.05) among all the samples. Compared with the corresponding samples of normal tissue, 204 spots showed a greater abundance and 209 showed a lower abundance in the SCC groups. These protein spots are indicated on the gel images shown in Figure 1.

**Figure 1:** Representative 2D-DIGE proteome map of lung cancer tissue samples vs. benign tissue samples. (A) Representative 2D-DIGE gel images. The extracted proteins were labeled with fluorescent dyes and separated by 2D-DIGE. (B) A representative two-dimensional gel image. A total of 1065 differentially expressed protein spots successfully identified by MALDI-TOF-MS are circled. (C) and (D): a mixture of all protein samples as the internal standard stained with Cy2 (blue). (E) and (F): adjacent normal tissues stained by Cy3 (green). (G) and (H): SCC tissues stained by Cy5 (red).

### Differential proteins identified by mass spectrometry

Among the 323 significantly altered spots detected by 2D-DIGE, 96 spots were judged to be valid and selected for further identification. Four of the 96 spots were identified by ESI-Q-TOF. Following a Mascot database search using the acquired MS data, 96 spots out of 81 proteins were identified as differentially expressed in cancer tissue as compared to benign tissue. Details of the experimental findings for protein identification, protein score, theoretical pI value, molecular weight, and average relative change are shown in Table 1.

**Table 1:** The list of differential proteins identified by MS.

Master No.	T test	Average Ratio	Protein ID	Protein name	Mascot Score	Gene Symbol	Gel MV (KD)/PI	Protein MW/PI
1	0.013	−1.66	Q14697	Neutral alpha-glucosidase AB	77	GANAB	87/5.4	107263/5.74
2	0.056	2.26	P14625	Endoplasmin	193	HSP90B1	90/4.3	92696/4.6
			P25686	DnaJ homolog subfamily B member 2	53	DNJB2		35672/5.61
			P59923	Zinc finger protein 445	58	ZN445		121282/10.44
3	0.0081	2.36	P55072	Transitional endoplasmic reticulum ATPase	91	VCP	85/4.7	89950/5.14
			Q969G7	Ankyrin repeat and SOCS box protein 1	72	ASB1		37732/8.55
4	0.05	5.05	P13645	Keratin, type I cytoskeletal 10	64	KRT10	85/6.2	59703/5.13
5	0.022	5.02	P13639	Elongation factor 2	65	EEF2	85/6.3	96246/6.41
6	0.0072	2.1	P55072	Transitional endoplasmic reticulum ATPase	80	VCP	83/4.8	89950/5.14
7	0.011	1.51	Q99798	Aconitate hydratase, mitochondrial	62	ACO2	80/6.4	86113/7.36
8	0.013	1.6	Q99798	Aconitate hydratase, mitochondrial	60	ACO2	80/6.5	86113/7.36
9	0.035	−2.76	P0C025	Putative nucleoside diphosphate-linked moiety X motif 17	59	NUD17	80/4.8	32598/6.4
10	0.03	−1.63	Q5TYW1	Zinc finger protein 658	48	ZNF658	75/4.9	125674/8.63
11	0.01	−1.63	P04217	Alpha-1B-glycoprotein	73	A1BG	80/4.7	54809/5.58
			Q3MIT2	Putative tRNA pseudouridine synthase Pus10	65	PUS10		60947/6.10
12	0.005	2.97	P11021	78 kDa glucose-regulated protein	200	HSPA5	80/4.5	72402/4.9
			Q6ZUX3	Protein FAM179A	54	F179A		111996/10.32
13	0.053	2.96	P11021	78 kDa glucose-regulated protein	81	HSPA5	80/4.5	72402/4.9
14	0.014	3.47	P11021	78 kDa glucose-regulated protein	267	HSPA5	80/4.6	72402/4.9
			O00291	Huntingtin-interacting protein 1	62	HIP1		
								117232/5.06
			Q6UWM7	Lactase-like protein	59	LCTLN		65560/8.87
			Q96N16	Janus kinase and microtubule-interacting protein 1	53	JAKMIP1		73506/5.77
15	0.016	1.62	P11142	Heat shock cognate 71 kDa protein	87	HSPA8	80/4.8	71082/5.2
16	0.059	−2.84	P02768.2	Serum albumin	140	ALB	70/5.3	71317/5.9
17	0.082	−2.74	P02768.2	Serum albumin	72	ALB	70/5.8	71317/5.9
18	0.038	−2.98	P02768	Serum albumin	267	ALB	70/5.3	71317/5.9
19	0.035	−3.74	P02768	Serum albumin	189	ALB	70/5.4	71317/5.9
20	0.067	−2.64	P02768.2	Serum albumin	117	ALB	70/5.2	71317/5.9
21	0.059	−3.51	P02768.2	Serum albumin	78	ALB	70/5.4	71317/5.9
22	0.011	−2.35	P04264	Keratin, type II cytoskeletal 1	60	KRT1	70/4.6	66149/8.16
23	0.0085	−2.45	P02768	Serum albumin	59	ALB	70/10	71317/5.92
24	0.05	1.88	P08107	Heat shock 70 kDa protein 1	190	HSPA1B	80/4.9	70294/5.4
25	0.026	−3.02	P02768	Serum albumin	364	ALB	70/5.6	71317/5.9
26	0.041	−2.79	P13645	Keratin, type I cytoskeletal 10	96	KRT10	70/3.2	59703/5.13
27	0.034	2.77	P11142	Heat shock cognate 71 kDa protein	178	HSPA8	75/6	71082/5.37
28	0.00027	1.8	Q13439	Golgin subfamily A member 4	64	GOLGA4	74/6	261892/5.33
29	0.057	−2.94	P02768.2	Serum albumin	91	ALB	68/5.4	71317/5.9
30	0.041	−2	P04040	Catalase	98	CAT	70/6.3	59947/6.9
31	0.0034	−2.62	Q8NCN4	RING finger protein 169	68	RNF169	67/4.6	78230/9.28
32	0.071	−1.83	P02768.2	Serum albumin	104	ALB	60/5.3	71317/5.9
33	0.0067	3.29	P10809	Heat shock protein 60	ESI-Q-TOF	HSPD1	63/4.8	61213/5.7
34	0.092	3.48	P23141.2	Liver carboxylesterase	82	CES1	60/5.8	62766/6.15
35	0.0058	4.61	Q9BQN1	Protein FAM83C	51	FAM83C	65/6	81540/9.2
36	0.0066	3.76	P35908	Keratin, type II cytoskeletal 2 epidermal	72	KRT2	65/6.4	66111/8.9
37	2.50E-05	4.66	P13647	Keratin, type II cytoskeletal 5	150	KRT5	65/6.2	62568/8.6
			P35908	Keratin, type II cytoskeletal 2 epidermal	51	KRT2		66111/8.85
38	0.035	2.08	P13645	Keratin, type I cytoskeletal 10	76	KRT10	65/6.2	59703/5
			P17030	Zinc finger protein 25	56	ZNF25		55050/10.11
39	0.061	3.83	Q9UMS4	pre-mRNA-processing fuetor19	ESI-Q-TOF	Prpf19	60/5.7	55180/6.14
40	0.1	2.7	P68371.1	Tubulin beta-2C chain;	185	TUBB2C	65/4.5	50255/4.79
41	0.024	3.53	P13645	Keratin, type I cytoskeletal 10	65	KRT10	65/6	59703/5
			P35908	Keratin, type II cytoskeletal 2 epidermal	52	KRT2		66111/8.85
42	0.027	3.77	P08670	Vimentin	83	VIM	60/4.6	53676/5.06
43	0.049	5.03	P14868	Aspartyc-tRNA synthetase, cytoplasmic	ESI-Q-TOF	DARS	60/5.8	57136/6.11
44	0.067	5.46	P05787.7	Keratin, type II cytoskeletal 8	56	KRT8	60/4.8	53671/5.52
45	0.018	16.32	Q8TDN1	Potassium voltage-gated channel subfamily G member 4	58	KCNG4	60/5.1	59797/6.23
46	0.021	14.23	P05787	Keratin, type II cytoskeletal 8	134	KRT8	60/5.2	53671/5.52
			Q6NVY7	Inositol monophosphatase 3	56	IMPAD1		38828/6.38
47	0.022	−2.16	P02675	Fibrinogen beta chain	53	FGB	64/5.9	56577/9.3
48	0.02	2.14	P08670	Vimentin	142	VIM	60/4.4	53676/4.9
49	0.045	2.93	Q9UBW7	Zinc finger MYM-type protein 2	67	ZMYM2	60/6.7	158403/5.9
			Q14532	Keratin, type I cuticular	59	KRT32		51769/4.7
50	0.03	2.22	P50454	Serpin H1	57	SERPINH1	60/8	46525/9.3
51	0.0066	2.01	Q6ZNA1	Zinc finger protein 836	60	ZNF836	62/6.2	111011/9.39
52	0.013	3.23	P06733	Alpha-enolase	112	ENO1	60/6.3	47481/7.01
			Q6ZNA1	Zinc finger protein 836	57	ZNF836		111011/9.39
53	0.06	32.55	P08670	vimentin	ESI-Q-TOF	VIM	60/4.3	53676/4.9
54	0.0052	3.61	Q04695	Keratin, type I cytoskeletal 17	243	KRT17	60/4.2	48361/4.97
55	0.023	3.05	Q15084	Protein disulfide-isomerase A6	62	PDIA6	60/4.3	48490/4.95
56	0.0067	−4.29	P08670	Vimentin	86	VIM	55/4.2	53676/4.9
57	0.024	−3.47	P08670	Vimentin	86	VIM	55/4.3	53676/4.9
58	0.058	1.91	P49411	Elongation factor Tu, mitochondrial	73	TUFM	55/6.1	49852/7.26
59	0.015	−6.49	P08670	Vimentin	88	VIM	55/4.3	53676/5.06
60	0.1	−17.08	P08670	Vimentin	76	VIM	55/4	53676/4.9
61	0.041	−1.69	Q9Y6G8	Estradiol 17-beta-dehydrogenase 12	57	HSD17B12	55/5.3	34416/9.34
62	0.022	1.8	O75874	Isocitrate dehydrogenase [NADP] cytoplasmic	61	IDH1	55/6.1	46915/6.53
63	0.033	−2.55	Q8IZC7.1	Zinc finger protein 101	65	ZNF101	55/5.5	51903/9.67
			P60709	Actin cytoplasmic 1	83	ACTB		42052/5.2
64	0.038	−1.67	P60709	Actin, cytoplasmic 1	62	ACTB	55/5.2	42052/5.29
65	0.013	2.67	Q8IZC7.1	Zinc finger protein 101	65	ZNF101	53/7	51903/9.67
66	0.017	−3.24	Q92889.3	DNA repair endonuclease XPF	62	ERCC4	53/4.9	105333/6.5
			Q8IZC7.1	Zinc finger protein 101	70	ZNF101		51903/9.67
67	0.038	−2.14	P60709	Actin, cytoplasmic 1	118	ACTB	50/4.8	42052/5.29
68	0.027	3.12	P04075	Fructose-bisphosphate aldolase A	86	ALDOA	58/7.2	39851/8.3
69	0.038	−4.75	Q9Y3P9	Rab GTPase-activating protein 1	6	RABGAP1	50/8	122915/5.15
			Q9BRK4	Leucine zipper putative tumor suppressor 2	49	LZTS2		73399/6.13
70	0.035	−2.01	P08727	Keratin, type I cytoskeletal 19	191	KRT19	52/4.2	44065/5.04
71	0.0039	1.86	P14550	Alcohol dehydrogenase [NADP+]	94	AKR1A1	48/6.1	36892/6.32
72	0.011	7.11	P04406	Glyceraldehyde-3-phosphate dehydrogenase	116	GAPDH	50/7	36201/9.3
73	0.0082	5.03	Q5S007.2	Leucine-rich repeat serine/threonine-protein kinase 2	68	LRRK2	48/8	289568/6.35
			Q14533.2	Keratin, type II cuticular Hb1	63	KRT81		56875/5.4
74	0.085	3.16	Q96PM5.1	RING finger and CHY zinc finger domain-containing protein 1	60	RCHY1	50/7.5	31743/6.3
75	0.012	−2.75	P07355.2	Annexin A2	96	ANXA2	45/6.7	38808/8.5
76	0.05	3.53	Q9BXF9	Tektin-3	63	TEKT3	45/7.4	57114/6.93
77	0.0075	−2.42	P08758.2	Annexin A5	102	ANXA5	40/4.4	35971/4.8
78	0.097	−2.2	Q16891	Mitochondrial inner membrane protein	64	IMMT	40/5	84025/6.08
			Q96DJ4	Tuberoinfundibular peptide of 39 residues	63	TIPF39		11195/11.83
79	0.043	−2.64	Q5H9K5	Zinc finger matrin-type protein 1	62	ZMAT1	40/5.3	75734/8.65
80	0.055	−3.26	Q96LU7	Uncharacterized protein C12orf28	72	C12orf28	38/7.5	31835/5.65
81	0.034	2.88	P63104	14-3-3 protein zeta/delta	110	YWHAZ	30/4.2	27899/4.73
82	0.025	−14.55	P02743	Serum amyloid P-component	105	APCS	30/5.1	25485/6.1
83	0.063	−2.47	P07288.2	Prostate-specific antigen	35	KLK3	30/4.7	29293/9
84	0.0081	2.67	P60174	Triosephosphate isomerase	132	TPI1	30/6.3	26938/6.45
85	0.01	−4.76	P02647	Apolipoprotein A-I	59	APOA1	20/5	30759/5.56
86	0.058	2.75	P09211.2	Glutathione S-transferase P	56	GSTP1	25/5	23569/5.3
87	0.075	8.11	P02792.2	Ferritin light chain	67	FTL	18/5	20064/5.4
88	0.014	3.34	P22392	Nucleoside diphosphate kinase B	62	Nme2	18/7	17401/8.52
89	0.052	−7.65	P68871	Hemoglobin subunit beta	40	HBD	13/7	16102/6.9
90	0.044	−4.8	P68871	Hemoglobin subunit beta	91	HBD	13/6.5	16102/6.9
91	0.082	−4.43	P68871	Hemoglobin subunit beta	94	HBD	13/6.3	16102/6.9
			Q13464.1	Rho-associated protein kinase 1	69	ROCK1		159102/5.58
92	0.065	−6.33	P68871	Hemoglobin subunit beta	59	HBD	12/6.7	16102/6.9
93	0.048	−5.84	P69905.2	Hemoglobin subunit alpha	64	HBA2	12/7.5	15305/9.4
94	0.093	−3.96	P69905.2	Hemoglobin subunit alpha	40	HBA2	12/7	15305/9.4
95	0.013	4.77	Q9Y2S2.3	L-gulonate 3-dehydrogenase; Gul3DH	60	CRYL1	11/7	35909/5.8
96	0.031	−3.19	Q6ZWJ1	Syntaxin-binding protein 4	60	STXBP4	10/5	62236/5.16

### Networks analysis of identified proteins by Ingenuity Pathway Analysis

A total of 81 proteins identified by mass spectrometry were analyzed by GO cluster analysis in the PANTHER database in terms of their cellular function, biological process, signal transduction pathway, cell component, and protein class, and a total of 74 proteins were identified in the database. For the category of biological process, the proteins were classified into groups consisting of cellular process, localization, transport, cellular component organization, apoptosis, system process, reproduction, response to stimulus, developmental process, generation of precursor metabolites and energy, metabolic process, cell cycle, immune system process, cell adhesion, and cell communication. For the category of protein class, the proteins classified into groups consisting of protease, cytoskeletal protein, transporter, transmembrane receptor regulatory/adaptor protein, transferase, oxidoreductase, lyase, ligase, nucleic acid binding, signaling molecule, enzyme modulator, defense/immunity protein, hydrolase, transfer/carrier protein, phosphatase, transcription factor, chaperone, structural protein, storage protein, isomerase, and receptor (Figure 2).

**Figure 2:** Classification of differentially expressed proteins according to their biological process and protein class. Pie charts display classification of the subset of differentially expressed proteins divided into 15 biological processes (A) and 21 protein classes (B). Molecular functions regulated by the differentially expressed proteins as classified by Gene Ontology.

### Validation of selected candidates by immunohistochemistry and western blot

Among the various proteins, two candidates were selected for further validation: (a) apolipoprotein A-1 (apoA1) and (b) serum amyloid P-component (SAP). The selected gel regions (spot 1957, apoA1 and spot 1854, SAP), and the quantification of these 2D spots are shown in Figure 3. The pI and MW of gel spot 1957 were 5.0 and 30 KD, respectively, and the spot was confirmed to be apoA1 by MALDI-TOF-MS. The pI and MW of apoA1 are 5.56 and 30.76 KD, respectively, which is consistent with the 2D gel position. The pI and MW of spot 1854 were 5.5 and 30 KD, and this spot was confirmed to be SAP by MALDI-TOF-MS. The pI and MW of SAP are 6.1 and 25.49 KD, respectively, which is consistent with the 2D gel position.

**Figure 3:** Detailed analyses of apoA1 and SAP by 2D-DIGE gel and MS. (A) 2D-DIGE gel images for apoA1 and SAP were labeled as 1957 and 1854. pI and MW for spot 1957 are 5.0 and 30 KD; pI and MW for spot 1854 are 5.5 and 30 KD. (B) and (D): Protein waves for spots 1957 and 1854 in 3-D view show both are single peaks, which signifies high protein content. (C) Comparison of congruity of spot 1957 in tumor and benign tissues of non-metastasis group (SqN) and metastasis group (SqM) shows similar results. Compared to expression in SqNP, expression in SqNT was down-regulated 4.76-fold, P = 0.01; Compared to expression in SqMP, expression in SqMT was down-regulated 5.2-fold, P = 0.019. (E) Comparison of congruity of spot 1854 in tumor and benign tissues of non-metastasis group (SqN) and metastasis group (SqM) shows similar results. Compared to expression in SqNP, expression in SqNT was down-regulated 14.55-fold, P = 0.0025; comparing to SqMP, expression in SqMT was down-regulated 3.72-fold, P = 0.041. (F) The Mascot Score of spot 1957 confirmed by MALDI-TOF-MS was 59. After hydrolysis of apoA1, the matching rate of peptides with the database was 14%. The matched peptides are shown in red (G) The Mascot Score of spot 1957 confirmed by MALDI-TOF-MS was 105. After hydrolysis of SAP, the matching rate of peptides with the database was 27%. The matched peptides are shown in red.

Western blot analyses showed low expression of both apoA1 (P = 0.033) and SAP (P = 0.001) in 20 pairs of SCC tissues, compared with adjacent normal tissue (Figure 4A), thereby confirming the 2D-DIGE data.

**Figure 4:** Expression of apoA1 and SAP in lung cancer and normal tissues. (A) Western blot analysis detected expression of apoA1 and SAP in 20 pairs of lung SCC and adjacent normal tissues. There was low expression of apoA1 and SAP in tumor tissues, and the differences in apoA1 and SAP expression in SCC and normal tissues were statistically significant, P = 0.033 and 0.001, respectively. (B) (a) Expression of apoA1 and SAP in normal tissue. Immunohistochemical analysis showed apoA1 and SAP as localized in the cell membrane and cytoplasm x200. (b and c) Expression of apoA1 and SAP in lung cancer tissues x200 and x400. Immunohistochemical analysis showed apoA1 and SAP were localized in the peripheral and central necrotic tissue of the cancer nest, but only slightly or not expressed in the cancer cells.

Immunohistochemical evaluation of 104 lung cancer tissues and 25 normal tissues revealed that the positive expression rates of apoA1 and SAP were 14.23% (15/104) and 9.62% (10/104), respectively, in cancer, and 84% (21/25) and 80% (20/25), respectively, in normal tissue (P<0.05) (Table 2 and 3). ApoA1 and SAP were localized in the cell membranes of the alveolar epithelial cells (Figure 4a), as well as the peripheral and central necrotic tissue of the cancer nest, but not in the cancer cells themselves, (Figures 4b, 4c), which signified low expression in lung cancer tissue. Statistical analysis indicated the expression levels of apoA1 and SAP were not associated with age, gender, differentiation, T stage, or clinical stage of the disease.

**Table 2:** Expression of SAP in lung cancer and normal tissues.

	SAP Expression			Positive rate (%)	P value
	(−)	(+)	(++)		
Lung cancer tissue	94	6	4	9.62	0.000
Normal tissue	5	2	18	80.00	

**Table 3:** Expression of apoA1 in lung cancer and normal tissues.

	apoA1 Expression			Positive rate (%)	P value
	(−)	(+)	(++)		
Lung cancer tissue	89	7	8	14.23	0.000
Normal tissue	4	5	16	84.00	

### Expression of apoA1 and SAP in serum of lung cancer patients

ApoA1 and SAP are secretory proteins, and can be detected in the serum. We used ELISA to detect the levels of apoA1 and SAP in blood serum from 150 lung cancer patients and 150 healthy subjects. The serum levels of apoA1 and SAP in lung cancer patients were 150.70±66.28 µg/mL and 632.00±229.42 ng/mL, respectively; for healthy subjects, the corresponding serum levels were 68.94±41.08 µg/mL and 209.39±127.87 ng/mL, respectively. These differences in apoA1 and SAP levels in the sera of lung cancer patients and healthy subjects were statistical significant (P<0.01) (Table 4, Figure 5).

**Figure 5:** Expression of apoA1 and SAP in sera of lung cancer patients and healthy donors.

**Table 4:** Expression of apoA1 and SAP in serum of lung cancer patients and healthy donors.

	n	apoA1 (µg/mL)	SAP (ng/mL)
Lung cancer patients	150	150.70±66.28	632.00±229.42
Healthy donors	150	68.94±41.08	209.39±127.87
P value		0.000	0.000

## Discussion

In this study, we performed a proteomic analysis of pulmonary SCC and adjacent normal tissues, with the goal of identifying new biomarkers for lung cancer. Compared to conventional 2DE, DIGE-based proteomics with fluorescence labeling has several advantages, including higher sensitivity, reproducibility over a linear dynamic range for better quantification, and fewer technical variations, because a pooled control is used as an internal standard.

Our proteomic data revealed 413 spots detected by 2D-DIGE that were altered in lung cancer tissue compared to benign tissue. Among these spots, 323 were significantly altered in their abundance (P≤0.05). Compared to the corresponding normal tissues, 204 spots were in higher abundance and 209 were at lower abundance in the SCC group. Among the significantly altered spots, 96 were judged to be valid and selected for further identification. Four of the 96 spots were identified by ESI-Q-TOF. Following a Mascot database search using the acquired MS data, 96 spots of 81 proteins were identified as differentially expressed in cancer compared to benign tissue. Based on criteria which included cellular function, biological process, signal transduction pathway, cell component, and protein class, 81 proteins identified by mass spectrometry were analyzed by GO cluster analysis in the PANTHER database.

Owing to the consistency of statistical results obtained from analyses of lung SCC and paired normal tissues (Paired T-test N, average ratio, Mascot Score, multipoint repetitive identification, protein functions, and bioinformatics analysis), we successfully identified several proteins that were definitely involved in cancer, including YWHAZ, TPI1, ROCK1, CAT, ENO1, VCR, VIM, GSTP, and ANXA2. In addition, in lung squamous carcinoma tissue, we revealed the presence of some proteins of unknown function that could be validated as potential biomarkers, including HSP90B1, HSPA8, HSPD1, HSPA5, DARS, GAPDH, EEF2, RCHY1, NME2, FGB, FTL, APOA1, STXBP4, HIP1, GOLGA4, SAP, ERCC4, RABGAP1, AKR1A, PRPF19, CES, KCNG4, ANXA5, UBB2C, ZNF101, ZMAT1, ALDOA, ALB, and HBD.This is the first report to confirm that the proteins DARS, HSP90B1, HSPA8, HSPA5, FGB, STXBP4, GOLGA4, ERCC4, RABGAP1, AKR1A, PRPF19, CES, KCNG4, ANXA5, TUBB2C, PDIA6, ZNF101, ZNF836, and ZMAT1 are related to lung tumorigenesis.

Furthermore, our bioinformatic analysis showed no results for the following proteins: ASB1, ZMYM2, CRYL1, C12 or f28, IMMT, TIPF39, RNF169, LRRK2, and NUD17. These may be new proteins of unknown function. It is known that most cancer cells exhibit increased glycolysis, and utilize this metabolic pathway for generation of ATP as a main source of energy. This phenomenon is known as the Warburg effect [15], and is considered as one of the most fundamental metabolic alterations which occur during malignant transformation. It is possible that GAPDH, ALDOA, and ENO1 may be involved in this process. Additionally, VIM and FGB were identified as proteins involved in epithelial-mesenchymal transition (EMT), and results of our follow-up experiments suggested that GAPDH, ALDOA, and eef-2 may also be involved in EMT.

Overall, our findings supplement current knowledge regarding the differential aspects of the lung cancer proteome, and facilitate the discovery of potential biomarkers.

Results of our analysis of the SCC proteome suggest that among the 81 proteins identified, serum amyloid P-component (SAP), apolipoprotein A1(apoA1), hemoglobin subunit beta (HBB), fructose-bisphosphate aldolase A (ALDOA), ferritin light (FTL), and huntingtin-interacting protein 1 (HIP1) are secretory proteins which can be easily detected in blood serum and may serve as biomarkers when screening for lung cancers. Based on factors including the average spot volume ratio, a spot's relative expression being changed by ≥1.5-fold (increase or decrease) by being associated with a non-malignant or malignant state, and the correlation between the proteins and tumorigenesis as determined by information retrieval, we found that SAP was down-regulated 14.55-fold in SqNT/SqNP, and 3.72-fold in SqMT/SqMP. In comparison, apoA1 was down-regulated 4.76-fold in SqNT/SqNP and 5.2-fold in SqMT/SqMP (Sq: squamous carcinoma; T: tumor; P: adjacent normal tissue; N: non-metastasis; M: metastasis). These differences of expression in tumor and adjacent normal tissue were statistically significant. ApoA1 is the major protein component of high-density lipoprotein (HDL) in plasma [16]. Studies conducted in vitro have confirmed that to satisfy the requirements for continuous proliferation, malignant tumor tissues contain increased amounts of cholesterol, and demonstrate greater activity of the rate limiting enzyme hydroxymethylglutaryl coenzyme A reductase (HMG-CoA reductase) [17]. We therefore speculate that apoA1 may play an important role in tumorigenesis. SAP is a highly preserved plasma protein synthesized by hepatocytes, and the major calcium-dependent specific DNA binding protein in blood serum. Jang JS. et al [18] searched proteome profiles of human stomach adenocarcinoma tissue and found that SAP activity was decreased. These results are similar to those in our research; however, we found no reports concerning screening of lung cancer tissues to investigate the possibility of utilizing these proteins as biomarkers. Therefore, we preferentially selected apoA1 and SAP for further research to determine their possible utility as biomarkers when screening for lung cancer.

In this study, only 7 cases of lung SCC were examined by 2D-DIGE for confirming the reliability of using apoA1 and SAP as biomarkers. We initially used western blot and IHC analysis to do the quantity and location study. The western blot results showed that apoA1 and SAP were down-regulated in lung squamous tissue, which was consistent with our 2D-DIGE results. The results of subsequent validation studies conducted using western blot and IHC methods demonstrated low expression of apoA1 and SAP in a significantly higher percentage of lung cancer tissues compared to corresponding benign tissues.

Additionally, we increased the sample size and investigated the expression of apoA1 and SAP in different types of lung cancer. Immunohistochemical evaluation of 104 lung cancer tissue sections and 25 sections of normal tissue revealed positive staining for apoA1 and SAP in the alveolar epithelium, but little or no positive staining in the cancer cells. Expression of apoA1 and SAP was not correlated with a histological classification of lung cancer, and we therefore believe that down-expression of apoA1 and SAP in lung cancer is nonspecific for squamous cell carcinoma. Our IHC study showed apoA1 and SAP were highly expressed in the peripheral and central necrotic tissue of the cancer nest, but only slightly or not expressed in the cancer cells. The western blot experiments were conducted using total protein extracts, and the results of IHC studies explain the high levels of apoA1 and SAP expression in some tumor tissues.

Our approach used to identify secretory proteins showed a significant differential expression of apoA1 and SAP in lung cancer patients and normal healthy tissue donors, which might be useful when utilizing these proteins as blood serum biomarkers for lung cancer. Because of this, the serum samples used in the preliminary validation study were obtained from 150 lung cancer patients and 150 healthy donors. Serum samples from cancer patients were obtained prior to surgery, and the patients had not received prior radiotherapy or chemotherapy; patients with hyperlipemia were also excluded. To minimize the influence of age, sex, and blood lipid abnormalities, negative control samples were obtained from age and sex-matched healthy donors. The differential expressions of apoA1 and SAP as determined by ELISA (Table 4) suggest that both apoA1 and SAP were highly expressed in samples of tumor tissue. There was a statistically significant difference (P<0.01) in the levels of apoA1 and SAP in the sera of cancer patients and normal subjects. Similar results were found for different types of lung cancer, and the results showed no relationship with histological classification of the tumor. Whereas expression of apoA1 and SAP was down-regulated in lung cancer as determined by 2D-DIGE, IHC, and western blot studies, the results showed divergence. We believe such divergence may be related to the excretion process of these proteins. Because they are secretory proteins, apoA1 and SAP can be secreted from tissue into the serum, which may lead to their reduced levels in tissue and increased levels in serum. This type of excretion process is a common phenomenon, and could explain the reason for divergence; however, additional studies should be conducted to confirm this hypothesis.

ApoA1 is synthesized in the liver and intestine as a prepro-protein. As a cofactor of lecithin-cholesterol acyltransferase (LCAT), apoA1 mediates a process known as “reverse cholesterol transport,” during which excess cholesterol from peripheral tissues is shuttled to the liver, converted to bile salts, and eventually excreted from the body. Previous reports concerning Apo have mainly focused on its role in cardiovascular and cerebrovascular diseases; however, we have recently demonstrated that tumors promote their rapid growth by acquiring and consuming as much nutrients and energy as possible [19]. The main biological function of lipids in vivo is energy storage. Such storage is closely related to tumorigenesis, and cancer patients tend to have high blood lipid levels [20]. SAP is a highly preserved plasma protein that is synthesized by hepatocytes. SAP is named for its ubiquitous presence in amyloid deposits, and is also a normal component of several basement membranes [21]. We speculate that the high levels of apoA1 and SAP in serum may be caused by their secretion by the liver and not secretion by tumor cells.

It has also been shown that certain tumor cells can synthesize acute phase proteins, such as IL6, to induce other cells to produce more apoA1 in inflammatory and cancer environments [22]. In our study, tissues from 104 cases of lung cancer and 25 normal subjects were subjected to IHC analysis, and we found that SAP and apoA1 showed low expression in tumor cells themselves, but high expression in central necrotic tissues of the cancer nest and peripheral necrotic tissues. These results may explain the high levels of apoA1 and SAP in the sera of cancer patients. Although the observed high levels of these proteins in the necrotic tissues could be artifacts due to non-specific staining, based on the literature, we cannot exclude the possibility that the necrotic tissues excrete more apoA1 and SAP, which could explain their high levels in sera.

Oram J Fet al [23] reported that because apoA1 is a main component of HDL, its levels are correlated with the presence of a tumor. Proliferating tumor cells require large amounts of cholesterol to form new cell membranes, and HDLs cannot maintain the equilibrium between intracellular and extracellular cholesterol. HDL binds to its cell surface receptors to promote the outflow of excess cholesterol, which leads to the low levels of cholesterol in cancer patients. Some studies have shown that apoA1 also plays a role in angiogenesis, which can contribute to the pathogenesis of cancer [24]. Yi ZF et al [25] found that a short 11-amino acid peptide (KV11) derived from apoA1 inhibits tumor growth by regulating cell migration and tumor angiogenesis by selectively blocking the VEGF-induced c-Src signaling pathway.

Some studies have reported the dysregulation of apoA1 and SAP during tumorigenesis. Bijon Chatterji et al [26] extracted proteins from the serum proteome of tumor bearing mice, separated them by 2-DE, and analyzed them using MALDI-TOF/TOF. They found that SAP was expressed during both the early and late stages of cancer. Park SY et al [27] used ESI-MS-MS to identify SAP in the plasma of rats with hepatic tumors, and confirmed the presence by western blot analysis. These results suggest that SAP might play an important role in the tumor progression. Jang JS. et al [18] searched the proteome profiles of human stomach adenocarcinoma tissue and paired surrounding normal tissue by MALDI-TOF, and found that SAP was decreased in tumor tissues. Our results obtained from analysis of clinical lung tumor tissues, combined with the published results described above, confirm the reliability of our data.

A method for serological monitoring of differentially expressed secretory proteins is of great value for tumor screening. In this study, we found that concentrations of apoA1 and SAP were higher in lung cancer patients than in healthy donors, and were not correlated with the histological classification or the grading system used for lung cancer. Therefore, we believe that patients with high levels of apoA1 and SAP in their blood serum may comprise a group at high risk for lung cancer. Our future study will further investigate the roles of apoA1 and SAP in lung tumorigenesis and the levels of apoA1 and SAP in the sera of a population at high risk for lung cancer, to establish criteria for medical surveillance.
